The article "Clinical Study on the Treatment of Benign Prostatic Hyperplasia by Embolization of Prostate Artery Based on Embosphere Microspheres and Gelatin Sponge Granules" was published in 2022. Journal: J Healthc Eng.

# Clinical Study on the Treatment of Benign Prostatic Hyperplasia by Embolization of Prostate Artery Based on Embosphere Microspheres and Gelatin Sponge Granules

**DOI:** 10.1155/2022/1424021

**Published:** 2022-01-25

**Authors:** Jinglei Liu, Dianwei Shi, Liang Li, Liming Cao, Jianyu Liu, Jingliang He, Zhihui Liang

**Affiliations:** ^1^Radiology Department, The 980 Hospital of PLA Logistic Force, Shijiazhuang 050082, Hebei, China; ^2^Tumor and Vascular Surgery Department, Anping People's Hospital, Hengshui 053600, Hebei, China

## Abstract

Prostatic hyperplasia can cause dysuria, such as frequent urination, urgency of urination, increased nocturia, poor urination, and other symptoms, which seriously affect the quality of life of old men. We aim to compare and analyze the safety and clinical effect of embolization of the target blood vessels of ruptured prostatic hyperplasia with gelatin sponge particles and embosphere microspheres. *Methods*. The transcatheter MRI was performed in 422 patients. Among them, 198 patients were treated with gelfoam particles and 224 patients were treated with embosphere microspheres. The clinical effect and adverse reactions were observed and analyzed by biochemical and imaging examination. Four hundred and twenty two cases were hemostasis. In the gelatin sponge group, 34 patients had recurrent bleeding 24–36 hours after embolization, 122 patients had different degrees of elevation of prostatic hyperplasia transaminase (31 cases increased to more than 1000 U/L), 198 patients had different degrees of elevation of bilirubin; in the microsphere group, there was no significant difference in prostatic hyperplasia function indexes between the two groups. *Conclusion*. Compared with the gelfoam embolic agent, the embosphere embolic microsphere has a good efficacy and safety in the treatment of prostatic hyperplasia rupture and hemorrhage, with a light adverse reaction, a low probability of recanalization, and little damage to the postoperative prostatic hyperplasia function, which is conducive to the benign recovery of perioperative patients and is worthy of clinical application.

## 1. Introduction

Prostatic hyperplasia is a common disease of old men. Its cause is that the dynamic and mechanical changes of the prostate have an oppressive effect on the bladder outlet and urethra, resulting in dysuria, such as frequent urination, urgency of urination, increased nocturia, poor urination, and other symptoms, which seriously affect the quality of life of old men [1–5]. Receptor blocker can reduce the tension of prostate and urethra smooth muscle [6–8]. Reductase inhibitor can reduce the volume of prostate by inhibiting the activity of 5 g reductase [9]. Benign prostatic hyperplasia (BPH) occurs since the cells of the prostate gland begin to multiply.

The article "Clinical Study on the Treatment of Benign Prostatic Hyperplasia by Embolization of Prostate Artery Based on Embosphere Microspheres and Gelatin Sponge Granules" was published in 2022. Journal: J Healthc Eng.

Embosphere microspheres have more advantages than traditional drugs. It is beneficial not only to improve the bioavailability and targeting of drugs but also to broaden the indications of original drugs. Gelatin sponge particles (GSPS) are absorbable particles. In previous studies, 6 GSPS with a diameter of 350–560 *µ*m has been used to treat liver metastasis of colorectal cancer and gastric cancer [10–13]. Clinically digital rectal examination, serum prostate-specific antigen (PSA), and transrectal MRI examination have different limits on the diagnosis and stage of abridged adenocarcinoma [14–16]. Compared with other techniques, MRI has the advantages of high resolution of soft tissue, multilevel imaging, and large field of vision. It is one of the best imaging methods for the diagnosis and staging of prostate cancer [17]. Therefore, we investigated the safety and clinical effect of embolization of the target blood vessels of ruptured prostatic hyperplasia with gelatin sponge particles and embosphere microspheres. Our opinion about this topic is that the embosphere embolic microsphere has a good efficacy and safety in the treatment of prostatic hyperplasia rupture and hemorrhage, with a light adverse reaction, a low probability of recanalization, and little damage to the postoperative prostatic hyperplasia function.

## 2. Materials and Methods

### 2.1. Study Object

A total of 422 patients (male 246 and female 176, age 31–81 years, average (60.0 Earth 21.0) years old) diagnosed as rupture and hemorrhage of prostatic hyperplasia in our hospital from September 2009 to December 2014 were collected. The patients had acute abdominal pain of different degrees, decreased blood pressure, with or without chest distress, pale complexion, cold sweat, and other shock symptoms. There were ascites of different degrees in percussion, and anticoagulant ascites and continuous decrease of hemoglobin were found in abdominal puncture. Among them, 78 cases were with tumor diameter <5 cm, 232 cases were with tumor diameter >5–10 cm, and 112 cases were with tumor diameter >10 cm. Child classification of prostatic hyperplasia function: 111 patients of Grade A, 213 patients of grade B, and 367 patients of grade C had blood pressure lower than 90 mmHg/60mmhg before treatment, of which 89 patients had hemorrhagic shock, shortness of breath, and severe confusion of consciousness. Four hundred and twenty two patients were divided into the gelatin sponge group (*n* = 198) and the microsphere group (*n* = 224).

### 2.2. Embolic Material

In the gelatin sponge group, the gelfoam particles' embolic agent of Hangzhou alikang Pharmaceutical Technology Co., Ltd. was used; in the microsphere group, the embosphere microspheres produced by biosphere medical Inc. of the United States were used as embolic agents.

The article "Clinical Study on the Treatment of Benign Prostatic Hyperplasia by Embolization of Prostate Artery Based on Embosphere Microspheres and Gelatin Sponge Granules" was published in 2022. Journal: J Healthc Eng.

### 2.3. Treatment

At the same time of pressor, antishock, and hemostasis, TAE was performed. After femoral artery puncture and intubation, hepatic arteriography was performed with 5frh catheter or 5F Cobra catheter (if necessary, angiography of diaphragmatic artery, splenic artery, and internal thoracic artery was performed to avoid blood supply of parasitic artery). The tumor distribution, tumor staining, blood supply, and signs of contrast agent overflow were observed to find the target blood vessel for bleeding. After diagnosis, the target blood vessel for bleeding was embolized with a microcatheter. In this study, both groups were treated with superselective catheterization to embolize the bleeding target vessels as much as possible. In the gelatin sponge group, an appropriate amount of gelatin sponge particles was injected for embolization, and in the microsphere group, embosphere embolization microspheres were injected for hemostasis until the bleeding artery was completely occluded and the casting had no reflow. After embolization, DSA confirmed that there was no clear sign of bleeding.

## 3. Results

### 3.1. Morphology of Embosphere Microspheres and Gelatin Sponge Particles

Figure 1 is a transmission electron micrograph of the embosphere microspheres by magnetic analysis and water washing. Composite microspheres are basically spherical with smooth surface and uniform particle size, with a diameter of about 122 nm. At the same time, we can clearly see that the black nanoparticle aggregates are coated in light-colored embosphere polymer microspheres, indicating that embosphere microspheres containing nanoparticles were successfully prepared by emulsion polymerization.  Figure 2 shows the perfect spherical shape of the typical gelatin sponge granules which indicates that embosphere microsphere microparticles with magnetic gaps are formed in emulsion polymerization.

### 3.2. Imaging Examination Results of Two Groups of Patients

In 422 patients with ruptured prostatic hyperplasia, after emergency hepatic artery embolization, the blood pressure of all the patients recovered and remained normal steadily on the day after operation, and the hemoglobin remained stable and did not drop again, indicating that hemostasis was effective.  Figure 3 shows MRI of massive prostatic hyperplasia in the right lobe with hemorrhage at the lower edge of the mass and the superselective intubation angiography showing hyperplasia, as can be seen from Figure 4. The statistic result is shown in Figure 5 (ALT and AST), and Figure 6 shows hemostatic prostatic hyperplasia function.

The article "Clinical Study on the Treatment of Benign Prostatic Hyperplasia by Embolization of Prostate Artery Based on Embosphere Microspheres and Gelatin Sponge Granules" was published in 2022. Journal: J Healthc Eng.

### 3.3. Comparison of the Degree of Benign Prostatic Hyperplasia between the Two Groups

The prostatic hyperplasia function was damaged in different degrees, and there was a significant difference between the indexes of prostatic hyperplasia function after operation and before operation. Among the 34 patients with recurrent bleeding 24–36 hours after embolization, 122 patients had different degrees of elevation of prostatic hyperplasia transaminase, and all patients had different degrees of elevation of bilirubin. In the microsphere group, blood pressure rose to the normal level after embolization, hemoglobin rose again and was stable, and there was no significant difference in prostatic hyperplasia function index between the two groups (Figure 7).

## 4. Discussion

In conclusion, embosphere microspheres may inhibit the expression of NF-*κ*B, then downregulate the expression of ICA M1, and inhibit the inflammatory response through its own antioxidation and free-radical scavenging properties [18, 19]. It also has a protective effect on the cerebral ischemia-reperfusion injury to a certain extent. Prostatic hyperplasia can also be seen with ruptured bleeding but relatively less. The treatment principle is to rescue shock, early diagnosis, and timely hemostasis [20]. The most common methods of hemostasis for patients with bleeding include comprehensive medical treatment, surgical operation, and TAE. Most patients will die of hemorrhagic shock. The hospital mortality rate is as high as 85%–100% [21–23]. However, most of the patients with ruptured and bleeding prostatic hyperplasia are in the middle and late stages, and most of them have severe cirrhosis at the same time [24]. They are generally in poor condition, accompanied with bloody ascites and even hemorrhagic shock. They cannot tolerate the re-trauma of general anesthesia and hepatectomy, and their resectability rate is very low. Most bleeding patients can only be treated with hemostasis such as simple packing and suture and ligation of hepatic artery [25, 26]. Severe prostatic hyperplasia function damage and jaundice can occur rapidly in perioperative period, and the patients finally died of prostatic hyperplasia failure. The perioperative mortality rate of prostatic hyperplasia rupture in surgical treatment is more than 60%. TAE, as a minimally invasive treatment, has become the first choice for the treatment of ruptured prostatic hyperplasia bleeding. It can identify the tumor by angiography [27].

The development and clinical application of microparticle embolic agents have greatly improved the medium- and long-term effect of TAE hemostasis. Particle embolic agents include gelatin sponge particles, embolic microspheres, and PVA. In the past, the commonly used embolic agents were gelatin sponge particles [28, 29]. A previous study also reported that lipiodol combined with gelatin sponge could embolize the blood vessels of ruptured prostatic hyperplasia in a short time [30].

The article "Clinical Study on the Treatment of Benign Prostatic Hyperplasia by Embolization of Prostate Artery Based on Embosphere Microspheres and Gelatin Sponge Granules" was published in 2022. Journal: J Healthc Eng.

## 5. Conclusion

In conclusion, TAE can effectively stop bleeding by superselective catheterization to the bleeding target artery. Different embolic agents will have different effects on the perioperative prostatic hyperplasia function. The embosphere microsphere particles have good efficacy and safety in the treatment of prostatic hyperplasia rupture and bleeding compared with the commonly used Gelfoam embolic agents. Because of its small expansion coefficient, long-term embolization, and the advantage of microcatheter injection, the adverse reactions of the patients are less, the probability of recanalization is lower, and the damage to the postoperative prostatic hyperplasia function is very little, which is beneficial to the benign recovery of the patients in the perioperative period, and it is worth popularizing in clinical application. However, there are still some limitations in our study. We still need to collect more diverse data and conduct more detailed and conductive results analysis.

## Figures and Tables

**Figure 1:** Morphology and features of embosphere microsphere.

**Figure 2:** Characterization of gelatin sponge particles.

**Figure 3:** MRI of massive prostatic hyperplasia in the right lobe with hemorrhage at the lower edge of the mass (arrow).

**Figure 4:** MRI of superselective intubation angiography showing hyperplasia (arrow).

**Figure 5:** Comparison of hemostatic prostatic hyperplasia function in two groups.

**Figure 6:** Comparison of hemostatic prostatic hyperplasia function in two groups: (1) HGB; (2) total bilirubin; (3) albumin.

**Figure 7:** Comparison of blood pressure, prostatic hyperplasia function, and hemoglobin before and after embolization and hemostasis in the microsphere group. (1) ALT (U/L); (2) BP (kPa); (3) AST (U/L); (4) HGB (g/L); (5) protein (g/L) umol/L

## Data Availability

The datasets used and/or analyzed during the current study are available from the corresponding author upon reasonable request.
